RETRACTED

# Measles-mumps-rubella vaccination timing and autism among young african american boys: a reanalysis of CDC data

**DOI:** 10.1186/2047-9158-3-16

**Published:** 2014-08-08

**Authors:** Brian S Hooker

**Affiliations:** 1 Simpson University, Redding, CA, USA

**Keywords:** Autism, Measles-mumps-rubella (MMR) vaccine

## Abstract

**Background:**

A significant number of children diagnosed with autism spectrum disorder suffer a loss of previously-acquired skills, suggesting neurodegeneration or a type of progressive encephalopathy with an etiological basis occurring after birth. The purpose of this study is to investigate the effectof the age at which children got their first Measles-Mumps-Rubella (MMR) vaccine on autism incidence. This is a reanalysis of the data set, obtained from the U.S. Centers for Disease Control and Protection (CDC), used for the Destefano et al. 2004 publication on the timing of the first MMR vaccine and autism diagnoses.

**Methods:**

The author embarked on the present study to evaluate whether a relationship exists between child age when the first MMR vaccine was administered among cases diagnosed with autism and controls born between 1986 through 1993 among school children in metropolitan Atlanta. The Pearson’s chi-squared method was used to assess relative risks of receiving an autism diagnosis within the total cohort as well as among different race and gender categories.

**Results:**

When comparing cases and controls receiving their first MMR vaccine before and after 36 months of age, there was a statistically significant increase in autism cases specifically among African American males who received the first MMR prior to 36 months of age. Relative risks for males in general and African American males were 1.69 (p=0.0138) and 3.36 (p=0.0019), respectively. Additionally, African American males showed an odds ratio of 1.73 (p=0.0200) for autism cases in children receiving their first MMR vaccine prior to 24 months of age versus 24 months of age and thereafter.

**Conclusions:**

The present study provides new epidemiologic evidence showing that African American males receiving the MMR vaccine prior to 24 months of age or 36 months of age are more likely to receive an autism diagnosis.

## Background

Autism is defined by persistent deficits in social communication and social interaction across multiple contexts and restricted, repetitive patterns of behavior, interests, or activities [1]. Autism incidence has risen dramatically over the past two decades [2] and it has recently been reported that one in sixty-eight children have this disorder [3]. In addition to these core deficits, autism has also been characterized by many other comorbid conditions including gastrointestinal issues, sleep issues, eating disorders and sensory processing issues [4].

RETRACTED

It has been estimated that as many as 62% of children with autism experience a period of regression during early childhood, characterized by loss of previously acquired skills [5]. This period has been reported as ranging between 6 and 36 months of age with the typical age of regression between 18 and 24 months [6]. This period of regression occurs within the same time period that children in the United States typically receive their required vaccinations and thus there have been many studies regarding the incidence of autism and the receipt of specific vaccines. One of the primary concerns has been the timing of the administration of the first measles-mumps-rubella (MMR) vaccine.

The relationship between the MMR vaccine and autism was first hypothesized by Wakefield et al. [7] in 1999 after the observation of a regressive phenotype of autism that appeared in general after the administration of the first MMR vaccine. Although several studies have affirmed such a relationship between the MMR vaccine and neurodevelopmental disorders including autism [8,9], many other studies purport no statistical relationship between the MMR vaccine and autism incidence. The latter studies have been performed using cohorts from Denmark [10], Japan [11] and Poland [12], as well as the MMR vaccine and pervasive developmental disorder in Canada [13]. In addition, in 2004, Destefano et al. [14] published a paper describing a case–control study completed on children, in metropolitan Atlanta, who had been born between 1986 and 1993. Within this study, the age at the first MMR vaccine was assessed as a factor in the incidence of autism. Using conditional logistic regression, with first MMR age as the independent variable and autism incidence as the dependent variable, the study authors assessed relative risk for obtaining an autism diagnosis for those children receiving the first MMR vaccine before and after 18 months, 24 months and 36 months of age. Destefano et al. [14] found a statistically significant relative risk of 1.49 (95% confidence interval [CI]: 1.04 – 2.14) at the 36 month cut-off (i.e., in a comparison of children receiving the MMR before versus after 36 months). Rather than concluding that the first MMR vaccine could be playing a causal role in autism in these children, the study authors instead attributed the increased risk to greater numbers of autistic children receiving timely vaccinations in order to participate in State of Georgia special education services.

In this paper, we present the results of a cohort study using the same data from the Destefano et al. [14] analysis. The focus of the current study is differences in results in specific gender and race groups.

RETRACTED

## Methods

### Cohort data

Cohort data were obtained directly as a “restricted access data set” from the Centers for Disease Control and Prevention (CDC) via a Data Use Agreement. Data were deidentified by the CDC in accordance with Family Education Rights and Privacy Act (FERPA) and the Health Insurance Portability and Accountability Act (HIPAA) prior to receipt by the study authors. Use of the CDC specifically for the study described herein was approved by the Simpson University Institutional Review Board, in accordance with U.S. Federal regulations.

### Study population

As reported by Destefano et al. [14] (CDC) in the original publication, “Children with autism were identified by the CDC from the Metropolitan Atlanta Developmental Disabilities Surveillance Program (MADDSP), a multiple-source, population-based surveillance program that monitors the occurrence of selected developmental disabilities among children in the 5-county metropolitan Atlanta area”. And further, “Autism cases were identified via screening and abstraction of source files at schools, hospitals, clinics, and specialty providers”. Of the cases identified, vaccination records were located for 660 children. Control children were chosen from “regular” education programs and were within the same age group and schools of attendance or neighboring school as cases. Children missing a vaccination form or with incomplete vaccination forms (where the forms did not list at least 1 diphtheria-tetanus-pertusussis vaccine by 2 years of age or at least 1 MMR vaccine at any age) were excluded from the study. Children with religious or medical exemptions were not excluded from the study. The listed exclusions yielded a cohort size of 624 cases and 1824 controls.

### Vaccination histories

Vaccination records were abstracted as described previously [14] from standardized state immunization forms that are required for all children who attend school and early intervention programs in Georgia.

### Demographic data

Demographic data including birthdate, gender and race were obtained for both case and control children via birth certificates or registration forms kept as a part of each child’s permanent school record. Georgia state birth certificate information was used to further obtain each child’s birthweight. Although actual birthweight data were not released by the CDC, case and control children were lumped into birthweight categories: under 1500 grams, between 1500 and 2500 grams and over 2500 grams. All individuals less than 3 years of age at the time of testing (1996) were excluded from the analysis.

RETRACTED

### Statistical analyses

The Pearson’s chi -squared test contained in the SAS® software was utilized for current statistical analyses, and a two-sided p-value < 0.05 was considered statistically significant. This is in contrast to the original Destefano et al. [14] (CDC) study, where a case–control study design was used, where 3 control children were matched to each case child, and analyzed using conditional logistic regression dichotomized for the three age cut-offs at 18, 24 and 36 months. Pearson’s chi-squared is, in general, a more conservative analysis and therefore chosen for the present study. However, our results were also confirmed using a conditional logistic regression design similar to the Destefano et al. [14] (CDC) study. In the present study, frequencies of cases were determined for first MMR ages of less than versus greater than 18 months, 24 months and 36 months in each separate analysis. When accounting for cases in the cohort that excluded low birth weight (<2500 g) African American children, it was necessary to report results at 31 months rather than 36 months in order to avoid reporting data from age categories or “cells” that possessed less than 5 individuals.

## Results

Table 1 shows the relationship between MMR timing and autism incidence for the entire cohort. As can be observed, there is a statistically significant effect for the cohort at 36 months (RR = 1.49, 95% CI: 1.04-2.14, p = 0.0289). However, this result appears to be caused by a stronger relationship (RR = 1.69, 95% CI: 1.11-2.57, p = 0.0138) seen exclusively in boys. Girls did not show any relationship between autism and MMR timing at any age group studied.

**Table 1:** Fisher’s exact analysis for the entire cohort

	**Total cohort**			**Males only**			**Females only**		
**Age cut-off**	**Relative risk**	**95% CI**	**p-value**	**Relative risk**	**95% CI**	**p-value**	**Relative risk**	**95% CI**	**p-value**
18 months	1.11	0.91-1.36	0.292	1.21	0.96-1.52	0.102	0.822	0.53-1.27	0.375
24 months	1.21	0.93-1.57	0.151	1.30	0.96-1.76	0.0826	0.936	0.54-1.62	0.812
36 months	1.49*	1.04-2.14	0.0289	1.69*	1.11-2.57	0.0138	0.996	0.49-2.04	0.992

*Result is statistically significant based on p < 0.05.

When looking specifically at African American children (Table 2), the relationship between MMR timing and autism incidence became more profound (RR = 2.30, 95% CI: 1.25-4.22, p = 0.0060) at 36 months of age. Again, this result was exclusively found in boys who showed statistically significant effects at both 24 months (RR = 1.73, 95% CI: 1.09-2.77, p = 0.0200) and 36 months (RR = 3.36, 95% CI: 1.50-7.51, p = 0.0019) of age. This effect again was not seen in females.

RETRACTED

**Table 2:** Fisher’s exact analysis for African American children only

	**Total cohort**			**Males only**			**Females only**		
**Age cut-off**	**Relative risk**	**95% CI**	**p-value**	**Relative risk**	**95% CI**	**p-value**	**Relative risk**	**95% CI**	**p-value**
18 months	1.24	0.90-1.70	0.184	1.36	0.95-1.95	0.0880	0.855	0.44-1.68	0.649
24 months	1.47	0.99-2.19	0.0562	1.73*	1.09-2.77	0.0200	0.861	0.40-1.88	0.707
36 months	2.30*	1.25-4.22	0.0060	3.36*	1.50-7.51	0.0019	1.01	0.38-2.68	0.982

*Result is statistically significant based on p < 0.05.

Table 3 shows results for the entire cohort excluding African American children. As can be observed, there is no statistically significant effect for any of the subclasses in either gender or age cut-off for MMR uptake. This shows that the effect observed overall is due to the very strong “signal” seen exclusively in African American boys. In other words, the strong, statistically significant relationship between younger first MMR age and higher autism incidence in African American males may be skewing the results for larger, more general populations that include African American males (e.g., all boys and all African Americans) to show a “relationship” that is actually only in African American males.

**Table 3:** Fisher’s exact analysis excluding African American children

	**Total cohort**			**Males only**			**Females only**		
Age cut-off	**Relative risk**	**95% CI**	**p-value**	**Relative risk**	**95% CI**	**p-value**	**Relative risk**	**95% CI**	**p-value**
18 months	1.06	0.81-1.38	0.668	1.17	0.87-1.58	0.309	0.734	0.41-1.31	0.292
24 months	1.06	0.75-1.50	0.745	1.10	0.74-1.62	0.642	0.910	0.41-2.00	0.814
36 months	1.13	0.72-1.78	0.588	1.19	0.72-1.97	0.490	0.835	0.28-2.48	0.745

Through investigating the cohort demographic data, it was found that there was a higher proportion of low birth weight African Americans compared to the entire cohort, specifically within the portion of the cohort that possessed a Georgia state birth certificate. The number of individuals with a birth weight under 2500 g for African Americans was 11.9% as compared to the total cohort at 8.66%. A final analysis was completed on African American children in the “birth certificate” cohort, excluding low birth weight individuals (Table 4). Results were obtained at 18 months, 24 months and 31 months, rather than 36 months, as there were insufficient cases (less than 5) at the 36 month mark to carry out the analysis. Even at 31 months, there were insufficient cases of African American females. Thus, these results are not included in the analysis. Even excluding low birth weigth individuals, a relationship was seen between first MMR age and autism incidence at 31 months for African American males (RR = 2.64, 95% CI: 1.08-6.46, p = 0.0280).

RETRACTED

**Table 4:** Fisher’s exact analysis for African American children excluding low birth weight

	**Total cohort**			**Males only**			**Females only**		
**Age cut-off**	**Relative risk**	**95% CI**	**p-value**	**Relative risk**	**95% CI**	**p-value**	**Relative risk**	**95% CI**	**p-value**
18 months	0.996	0.66-1.51	0.986	1.06	0.66-1.69	0.819	0.804	0.32-2.00	0.637
24 months	1.29	0.76-2.21	0.348	1.53	0.82-2.85	0.178	0.731	0.25-2.14	0.567
31 months*	1.85	0.91-3.79	0.0872	2.64	1.08-6.46	0.0280	---	---	---

*31 month cut-off was used as 36-months yielded results for African American males with <5 individuals per cell in the analysis.

## Discussion

The results show a strong relationship between child age at the administration of the first MMR and autism incidence exclusively for African American boys which could indicate a role of the vaccine in the etiology of autism within this population group. This particular analysis was not completed in the original Destefano et al. [14] (CDC) study. Although the previous study considered MMR timing and African Americans in general, no statistically significant effect was observed. This is in contrast to our result for African Americans in general, because the CDC study limited the total African American cohort to include only those individuals who possessed a valid State of Georgia birth certificate which decreased the statistical power of their analysis. Although a statistically significant relationship between first MMR age and autism incidence was seen in the general (all races) population within the earlier Destefano et al. [14] study, the coauthors interpreted this result as an artifact of “healthcare seeking behavior” citing that autistic children would receive their vaccines earlier in order to enroll in State of Georgia early intervention programs. However, it is highly unlikely that this type of behavior would be seen exclusively in African American males and thus, alternative hypotheses must be explored, including the possibility that the MMR vaccine may be causally linked to autism in African American males.

It should be noted that a recent publication has shown that the prevalence of autism in African Americans is nearly 25% higher than that of whites [15]. This value was obtained when CDC data were appropriately analyzed based on socioeconomic status. This could be due to issues regarding vitamin D status with African Americans as it has been estimated that vitamin D sufficiency among whites is between 30-60% but is only 5-10% among African Americans [16]. Patrick et al. [17] have very recently proposed a mechanism for the link between vitamin D status and autism via selective production of serotonin in the brain. Disruption of the serotonergic system is a very consistent observation with autism [18] as serotonin promotes prosocial behavior and proper assessment of emotional social cues [19].

RETRACTED

Vitamin D has a multitude of other physiological functions in vivo. Vitamin D receptor has been found in many different tissues including the small intestine, colon, osteoblasts, activated T and B lymphocytes, islet cells and most organs in the body [20]. Vitamin D has also been implicated in many important physiological processing including modulation of activated T and B lymphocyte function [21,22] and prevention of inflammatory bowel disease [23]. Lower vitamin D status African American females are more susceptible to lupus [24]. Also, Epstein-Barr Virus antibody titers are significantly higher in African American youth as compared to compared to white youth [25] which may be a consequence of vitamin D insufficiency. Also, childhood adversity, which could be more prevalent in African American boys, can have lasting immune consequences [26].

Gallagher et al. [27] have reported previously regarding the Hepatitis B vaccine and autism in neonates, specifically within the 1997 to 2002 time period when this vaccine series still contained thimerosal. Regarding non-whites they specifically stated in the abstract, “Non-white boys bore greater risk” of receiving an autism diagnosis if they received the Hep B as neonates. The data reported in this paper show a statistically significant risk ratio of 5.53 (p = 0.019) for black boys as opposed to white boys who had a risk of 1.87 (p = 0.171) which was not statistically significant, when looking at autism in those infants that received their first Hep B vaccine during the first month of life.

A strength of the current study is that the MADDSP data were collected independently of the design used in the analysis. These data were collected as part of the diagnoses individuals received as part of their participation in special education program and as such, the healthcare providers in no way were thinking about the potential association between vaccine exposures and potential health outcomes. Also the current study controlled for a possible association between low birth weight individuals and autism as in the final analysis on the African American cohort, all children of birthweight less than 2500 grams were eliminated from the cohort. Although low birthweight (LBW) has been shown to be associated with an increased risk of autism [28], insufficient information existed within the study population to assess the effect of LBW on autism incidence or any interaction between LBW and MMR timing.

RETRACTED

The weaknesses of the current study include the age groups selected for autism cases and controls within the original data set. The average age to receive an autism diagnosis has been reported (using the CDC’s Vaccine Safety Datalink) as between 3.7 [29] and 4.2 years of age [30]. However, the CDC’s dataset included controls as young as 3 years of age who could have been “too young” to receive an autism diagnosis. Accordingly, there is a greater than 50% probability that some of the controls could have later received an autism diagnoses, thus skewing the analysis to the null (“no effect”) hypothesis. However, when the analysis was recompleted using controls that were six years of age or older, very similar results were obtained (data not shown). Also, information on the timing of other infant vaccines was not released by the CDC and thus it was impossible to control this factor in the current analysis. In addition, socioeconomic factors were not assessed in the current analysis. Thus, any differences in “healthcare seeking behavior” among individuals vaccinated ontime versus late could not be assessed.

## Conclusions

The present study provides new evidence of a statistically significant relationship between the timing of the first MMR vaccine and autism incidence in African American males. Using a straight-forward, Pearson’s chi-squared analysis on the cohort used in the Destefano et al. [14] (CDC) study, timing of the first MMR vaccine before and after 24 months of age and 36 months of age showed relative risks for autism diagnoses of 1.73 and 3.36, respectively. Future studies should be completed to further evaluate the relationship of first MMR timing and neurodevelopmental maladies, including autism, especially in underserved populations.

Routine childhood vaccination is considered an important public health tool in reducing the morbidity and mortality associated with infectious diseases. However, consideration should be made in the current United States vaccination schedule for genetic subpopulations that may be associated with vaccine adverse events. Additional research is required to better understand the relationship between MMR exposure and autism in African American males.

## Abbreviations

CDC: Centers for Disease Control and Prevention; CI: Confidence Interval; Hep B: Hepatitis B vaccine; MADDSP: Metropolitan Atlanta Developmental Disabilities Surveillance Program; MMR: measles-mumps-rubella vaccine; RR: Relative Risk.

## Competing interests

Dr. Hooker has been involved in vaccine/biologic litigation.

## Authors’ contributions

BH was the main manuscript writer and computer programmer.
